This article has been retracted.

# Obesity-induced adipokine imbalance impairs mouse pulmonary vascular endothelial function and primes the lung for injury

**DOI:** 10.1038/srep11362

**Published:** 2015-06-12

**Authors:** Dilip Shah, Freddy Romero, Michelle Duong, Nadan Wang, Bishnuhari Paudyal, Benjamin T. Suratt, Caleb B. Kallen, Jianxin Sun, Ying Zhu, Kenneth Walsh, Ross Summer

**Affiliations:** 1 Center for Translational Medicine and Jane and Leonard Korman Lung Center, Thomas Jefferson University, Philadelphia, PA 19107, USA; 2 Department of Radiology, Thomas Jefferson University, Philadelphia, PA 19107, USA; 3 Department of Medicine, University of Vermont College of Medicine, Burlington, VT 05405, USA; 4 Department of Obstetrics and Gynecology, Thomas Jefferson University, Philadelphia, Pennsylvania 19107, USA; 5 Department of Respiratory Medicine, Changhai Hospital, Second Military Medical University, Shanghai, China; 6 Whitaker Cardiovascular Institute, Boston University School of Medicine, Boston, MA, 02118, USA

## Abstract

Obesity is a risk factor for the development of acute respiratory distress syndrome (ARDS) but mechanisms mediating this association are unknown. While obesity is known to impair systemic blood vessel function, and predisposes to systemic vascular diseases, its effects on the pulmonary circulation are largely unknown. We hypothesized that the chronic low grade inflammation of obesity impairs pulmonary vascular homeostasis and primes the lung for acute injury. The lung endothelium from obese mice expressed higher levels of leukocyte adhesion markers and lower levels of cell-cell junctional proteins when compared to lean mice. We tested whether systemic factors are responsible for these alterations in the pulmonary endothelium; treatment of primary lung endothelial cells with obese serum enhanced the expression of adhesion proteins and reduced the expression of endothelial junctional proteins when compared to lean serum. Alterations in pulmonary endothelial cells observed in obese mice were associated with enhanced susceptibility to LPS-induced lung injury. Restoring serum adiponectin levels reversed the effects of obesity on the lung endothelium and attenuated susceptibility to acute injury. Our work indicates that obesity impairs pulmonary vascular homeostasis and enhances susceptibility to acute injury and provides mechanistic insight into the increased prevalence of ARDS in obese humans.

It is now firmly established that obesity contributes to the development of cardiovascular morbidity and mortality from conditions including hypertension, coronary artery disease, and stroke^1^,^2^. Although the mechanisms by which obesity impairs vascular tissue functions are complex and not fully elucidated it is generally accepted that chronic low-grade systemic inflammation plays a role in promoting disease^3^. This chronic low-grade systemic inflammation results from a combination of factors including elevated lipid levels and altered production of pro- and anti-inflammatory factors (i.e. adipocytokines) by the expanded and altered adipose tissue^4^.

Although the pulmonary circulation is physically connected to the systemic circulation and is exposed to identical circulating factors, it cannot be assumed that the vasculature in each tissue responds in the same ways to diverse cues. In fact, endothelial functions vary between tissues (consider the blood-brain barrier or the blood testis barrier) and surprisingly little is known about the effects of obesity on pulmonary vascular function^5^. Important differences between the systemic and pulmonary vasculatures exist, including the fact that the pulmonary vasculature is a low pressure system while the systemic vasculature is a high pressure system, and the fact that the pulmonary vasculature vasodilates rather than vasoconstricts in response to hypoxia. Pressure and other features of blood flow are known to affect tissue functions and may, in part, explain why certain vascular diseases (i.e. atherosclerosis, essential hypertension) do not affect the pulmonary circulation^6^,^7^,^8^,^9^. Whether obesity-related factors affect the pulmonary vasculature in the same ways that they affect the systemic vasculature remains largely unknown.

While clinical studies have yet to establish whether the prevalence of pulmonary vascular diseases such as pulmonary arterial hypertension are increased in obese individuals, emerging evidence suggests that obesity is a risk factor for the development of acute respiratory distress syndrome (ARDS)^10^,^11^,^12^. ARDS is a severe inflammatory lung condition that develops abruptly in vulnerable patients with co-morbidities such as pneumonia, sepsis, or pancreatitis. Although ARDS is not ordinarily classified as a pulmonary vascular disease, hallmark features of this condition include widespread immune activation of the lung endothelium and loss of endothelial cell barrier functions^13^,^14^. Given that ARDS is, ultimately, a disorder of vascular function, we hypothesized that obesity-related factors may adversely affect the pulmonary vasculature rendering obese individuals more susceptible to ARDS.

While little is known about the effects of obesity on pulmonary vascular homeostasis, studies using adiponectin-deficient mice provide insight into the interaction between adipose tissue and the pulmonary circulation^15^,^16^. Adiponectin, an adipose tissue-derived hormone, exhibits anti-inflammatory and vascular protective properties, and its levels decrease with increasing fat mass^17^,^18^. Because hypoadiponectinemia is a feature of the obese state, mice deficient in this hormone are commonly used as a tool for modeling the obese condition. However, very few, if any, studies evaluate the role of this adipokine within the complex mileau of the obese organism. Recently, mice with targeted deletion of the adiponectin gene were noted to develop spontaneous activation of their lung endothelium and to exhibit enhanced susceptibility to acute lung injury (ALI), the murine equivalent of ARDS^16^. Moreover, restoring serum adiponectin levels in these metabolically-normal mice decreased their susceptibility to ALI, at least in part, by suppressing the expression of lung endothelial cell adhesion markers and decreasing the severity of pulmonary vascular leak after LPS administration^16^. While adiponectin deficient mice do not reflect the complex physiology of obesity, the above studies provoked our central hypothesis, namely that obesity disrupts pulmonary vascular homeostasis thereby contributing to the onset of inflammatory vascular diseases in the lung. In this study, we tested this hypothesis in mouse models of diet-induced obesity and studied the mechanisms underlying the observed effects of obesity on pulmonary injury.

## Results

### Obesity alters expression of cell adhesion molecules in pulmonary vascular endothelium

To study the effects of obesity on vascular homeostasis we first fed AKR/J and DBA/2J mice a high fat diet or standard chow for a total of 14 weeks. These strains of mice were selected for their ability to maintain normal glucose control when obese, thus minimizing the effects of hyperglycemia in our model system^19^. As shown in supplemental table 1, we found that mice fed the high fat diet exhibited significantly more weight gain compared to standard chow-fed mice. Moreover, mice on the high fat diet displayed normal fasting blood glucose levels and minimal elevations in serum glucose after intraperitoneal glucose challenge.

To determine whether obesity impairs vascular function in our model system we measured soluble E-selectin levels in the circulation of lean and obese mice. E-selectin is an endothelial-specific adhesion marker whose serum concentration increases in response to vascular injury. We found that serum E-selectin levels were significantly increased in the obese state in AKR/J (Fig. 1a) and DBA/2J (Supplementary Fig. 1a) mice when compared to lean controls. To assess whether increases in serum E-selectin were representative of changes within the pulmonary circulation we evaluated the expression of vascular adhesion markers in the lungs of lean and obese mice. Consistent with injury to the lung endothelium, we found that transcript and protein levels for E-selectin, ICAM-1 and VCAM-1 were significantly increased in whole lung and in freshly isolated lung endothelial cells from AKR/J (Fig. 1b–d) and DBA/2J (Supplementary Fig. 1 b,c) obese mice.

Because endothelial barrier function is often disrupted when vascular adhesion markers are upregulated, we hypothesized that obesity might also modify the expression of structural proteins important in maintaining vascular integrity. Consistent with this hypothesis, we found that pulmonary endothelial junctional adherens proteins VE-cadherin and β-Catenin were decreased and phosphorylated Src (pSrc) was significantly increased in the lungs of obese mice when compared to lean controls (Fig. 1e & Supplementary Fig. 1d). Importantly, these changes in the expression of junctional adherens proteins were not associated with the spontaneous development of pulmonary edema as assessed by lung histology (data not shown), Evan’s blue dye accumulation or BAL fluid protein concentration (Fig. 1f,g). These findings indicate that, despite the measured changes in pulmonary vascular junctional adherens proteins, the lung endothelium of obese mice is capable of maintaining its barrier functions in the unchallenged state.

### Serum from obese mice alters expression of adhesion markers and junctional adherens in isolated lung endothelial cells

Because chronic inflammation has been implicated in the pathogenesis of blood vessel dysfunction in the systemic vasculature of obese individuals^20^, we reasoned that systemic inflammation might similarly contribute to the pathological effects we observed in the pulmonary vasculature of obese mice. As expected, our obese mice demonstrated elevated levels of circulating leptin, free fatty acids, triglycerides, and cholesterol and lower levels of the anti-inflammatory hormone adiponectin (Fig. 2a–e & Supplementary Fig. 2a–d) when compared to lean mice. To determine whether alterations in serum factors contribute to the observed gene expression changes in the pulmonary vasculature of obese mice, we cultured primary lung microvascular endothelial cells with serum from lean or obese mice and measured the expression of adhesion markers and endothelial junctional proteins. As show in fig. 2f,g, we found that lung endothelial cells cultured with serum from obese mice exhibited a significant increase in the expression of E-selectin, ICAM-1 and VCAM-1 and a marked decrease in the expression of VE-cadherin and β-Catenin as well as an increase in pSrc. These findings indicate that the obese endocrine milieu impairs pulmonary vascular endothelial gene expression similar to its effects on the systemic vasculature.

### Obesity exacerbates LPS-induced lung inflammation and vascular injury

To assess whether changes in endothelial junctional adherens proteins in the lungs of obese mice influences the susceptibility of the pulmonary vasculature to injury, we instilled LPS into the tracheal lumen of lean and obese mice. Single dose LPS treatment is a model of acute lung injury that recapitulates many features of human ARDS including massive immune cell infiltration, enhanced production of pro-inflammatory factors, and the loss of vascular integrity^21^. As shown in Fig. 3 & Supplementary Fig. 3, we detected a robust inflammatory response in all mice after LPS administration, but the severity of inflammation was increased in the obese mice. We found that airspace and tissue neutrophilia, as well as levels of chemotactic factors (KC and MIP2) and pro-inflammatory cytokines (TNF-α and IL-6), were markedly increased in the lungs of LPS-injured obese mice when compared to lean mice (Fig. 3a–g & Supplementary Fig. 3a**-**f). Additionally, we found that obese mice developed more vascular injury after LPS instillation, manifested by upregulation of ICAM-1, VCAM-1 and E-selectin, downregulation in the expression of VE-cadherin and β-Catenin, and increased expression of pSrc (Fig. 4a–c & Supplementary Fig. 4a-c) Further, we also found that endothelial barrier function was reduced in the lungs of obese mice as evident by increased peri-vascular fluid surrounding pulmonary blood vessels, higher lung wet/dry ratio, increased Evans blue extravasation into the lung and higher protein concentration (total protein and IgM) in the BAL fluid from obese mice (Fig. 4d–h & Supplementary Fig. 4d,e). Taken together, these findings indicate that obesity enhances susceptibility to acute lung injury by augmenting inflammation and disrupting endothelial cell barrier functions.

### Cardiovascular function is preserved in obese mice during ALI

Because obesity is known to impair cardiac function^22^, we hypothesized that left ventricle dysfunction might contribute to enhanced vascular permeability in the lungs of obese mice after LPS administration. To test this hypothesis, we performed transthoracic echocardiography to assess left ventricular systolic function in lean and obese mice at baseline and at 4 h after LPS administration. The 4 h time point was selected because our prior work indicated that vascular leak is a prominent feature of the LPS-injured lung by this time point^23^. As shown in Supplementary Table 2, we did not observe significant differences in left ventricular function, as measured by ejection fraction or percent fractional shortening, in lean or obese mice after LPS treatment. Consistent with these data, we found that hemodynamic parameters measured during invasive monitoring; including heart rate, blood pressure, central venous pressure and both right and left ventricular change in pressure over time (dp/dt) were not significantly different between lean and obese mice at baseline or after injury (Supplementary Table 3). Taken together, these findings indicate that cardiac function is largely preserved in our model system and suggest that intrinsic defects within the lung endothelium contribute most significantly to the development of pulmonary edema after LPS administration.

### Adiponectin protects against LPS-induced lung injury in obese mice

We previously demonstrated that restoring serum adiponectin levels in metabolically-normal adiponectin-deficient mice attenuates LPS-induced acute lung injury^16^. Because adiponectin deficiency represents only one aspect of the obese state we sought to test whether adiponectin repletion is sufficient to protect the LPS-treated lung in the complex milieu of the obese state. Thus, we compared adiponectin deficient and adiponectin-replete obese mice after 14 weeks of high-fat diet. We demonstrated that adiponectin gene therapy was effective in restoring peripheral adiponectin levels at 1 and 3 days after treatment (Fig. 5a and data not shown). Restoration of adiponectin levels in obese mice was associated with marked reductions in serum free fatty acids, triglycerides and leptin levels in the serum (Fig. 5b–d).

We tested whether restoring serum adiponectin levels modifies the effects of obesity on the pulmonary vasculature. First, we evaluated the expression of vascular adhesion markers in the lungs of obese control mice and obese mice on day 3 after repletion of adiponectin levels. We found that expression of E-selectin, ICAM-1 and VCAM-1 were significantly decreased in the lungs of obese mice after repletion of adiponectin (Fig. 5e). This decrease in adhesion markers was associated with an increase in the expression of endothelial junctional proteins VE-cadherin, β-Catenin and a decrease in expression of pSrc (Fig. 5f), indicating that adiponectin effectively reversed the deleterious effects of obesity on the lung endothelium *in vivo*. We next determined whether adiponectin repletion alters the susceptibility of obese mice to acute lung injury; we measured inflammatory and injury responses to LPS in control and adiponectin-replete obese mice. Adiponectin-replete mice exhibited significantly less lung inflammation than control mice as demonstrated by decreased TNFα expression and reduced pulmonary immune cell infiltration measured 24 h after LPS administration (Fig. 6a–c). The observed reduction in lung inflammation was associated with a marked attenuation of vascular injury in the adiponectin-replete obese mice. We observed reduced expression of vascular adhesion markers, an increase in expression of endothelial junctional adherens proteins, decreased pSrc and peri-vascular edema, and reduced protein accumulation in the BAL fluid after LPS instillation (Fig. 6d–h). These findings indicate that adiponectin reverses the endothelial cell phenotypic changes associated with obesity and reduces susceptibility of obese mice to acute lung injury.

## Discussion

We hypothesized that obesity alters pulmonary vascular endothelial functions similar to its effects in the systemic vasculature. We tested whether obesity renders lungs more vulnerable to injury in a mouse model system of ALI/ARDS. We have shown that obesity exerts deleterious effects on the pulmonary vasculature by disrupting the expression of endothelial junctional adherens proteins and enhancing the expression of adhesion molecules in two mouse strains. These perturbations are associated with an increase in the susceptibility of the pulmonary vasculature to injury. Further, our mechanistic studies indicate that systemic inflammation participates in the barrier and immune changes observed in the lung endothelium of obese mice, and we show that restoring serum adiponectin levels in obese mice reverses pathological changes in the lung endothelium and attenuates the susceptibility to developing ALI. These data complement our prior study that investigated ALI in adiponectin-deficient mice^16^. Taken together, we conclude that adiponectin is both essential and sufficient in controlling key processes that contribute to ARDS in experimental systems.

In many cases, including aspiration and infectious pneumonias, upregulated vascular adhesion markers and reduced expression of endothelium junctional adherens proteins is associated with increased vascular permeability and enhanced leukocyte transmigration from the intravascular space into lung parenchyma^24^,^25^. However, these histopathological features are noticeably absent from the lungs of obese mice in our model system. These findings imply that, at baseline, the obese lung endothelium retains adequate barrier function despite being poised to respond poorly to insult. While we recognize that more subtle changes in the lung architecture such as mild interstitial edema or margination of leukocytes along blood vessel walls have not been excluded, these types of findings would require more sophisticated histological analyses then were pursued in our studies.

Although endothelial barrier function is preserved in the lungs of obese mice at baseline we found that the obese state markedly increased vascular permeability in response to LPS administration. This enhanced susceptibility to injury is consistent with findings in human studies demonstrating that endothelial-specific injury markers (i.e. Von Willebrands factor) are increased in the serum of obese patients with ARDS when compared to their lean counterparts^26^. While findings in this study suggest that enhanced vascular leak resulted primarily from structural changes within the lung endothelium of obese mice we cannot exclude the possibility that the integrity of the lung’s epithelium might also be impaired in obese mice. Future studies examining the effects of obesity on lung epithelial barrier function will be important for understanding why obese individuals are more susceptible to developing ARDS.

Another important finding in our study is the observation that neutrophil influx is significantly increased in lungs of obese mice after LPS administration. One logical explanation for these findings is that neutrophil recruitment is facilitated by the increased expression of vascular adhesion markers and the reduced expression of junctional adherens proteins in the lung endothelium of obese mice^27^,^28^,^29^. Moreover, we postulate that serum mediators flooding the distal airspaces of the lung after injury may also act to directly promote neutrophil recruitment (e.g. leptin) or enhance the production of neutrophil chemotactic factors. This mechanism might explain why we found that neutrophil chemotactic factors MIP2 and KC were increased in the lungs of obese mice after LPS administration^30^,^31^. Additionally, it is likely that baseline increases in circulating neutrophils, which is well-documented in obesity, and was confirmed in our model system (Supplementary Table 4), might have contributed to the enhanced leukocyte influx to the lung after injury.

While our study focused primarily on the pulmonary vasculature, we recognize that obesity may affect additional cell types within the lung including epithelial and immune cell types. Since obesity is known to alter the behavior of macrophages (promoting the shift to an M1 pro-inflammatory phenotype) in other tissues (e.g. adipose tissue) we postulate whether alveolar macrophage functions might also be altered in the obese lung^32^,^33^. Although we did not detect differences in the number of alveolar macrophages in BAL fluid (Fig. 3a) in lean and obese mice we cannot exclude the possibility that functional differences exist between these populations. Enhanced M1 macrophage polarization could possibly explain why we observed an increase in TNFα and IL-6 in the lungs of obese mice after LPS administration^34^.

Studies in humans indicate that obesity predisposes to the development of ARDS. Somewhat surprisingly, diabetes mellitus (T2DM) confers protection against the development of ARDS^35^,^36^. It has been proposed that the mitigating effects of diabetes are related to the immune suppressive effects observed in this condition; specifically, diabetes is known to impair neutrophil functions including chemotaxis, phagocytosis, cell adhesion and oxidative burst^37^. Our studies minimized the potentially confounding effects of hyperglycermia/diabetes and obesity by employing mouse models that maintain normal insulin sensitivity while obese. The failure to account for the effects of hyperglycemia/diabetes may explain why recent studies using diabetes-prone C57Bl/6 or db/db mice found that susceptibility to acute lung injury was attenuated in their model systems^37^,^38^. These groups observed a blunted neutrophil chemotactic response in their obese mice. While we recognize that other factors are likely to contribute to strain-specific differences in the susceptibility of obese mice to developing ALI, moving forward, it will be important to distinguish between the effects of obesity and diabetes in each model system.

We have studied three distinct models of hypoadiponectinemia (adiponectin deficient mice and two strains of diet-induced obese mice), each of which is more susceptible to developing ALI than the wild-type/lean mouse. Interestingly, we also observed that diet-induced obese mice on the C57Bl/6 background, which are not more susceptible to developing ALI, neither develop hypoadiponectinemia nor exhibit phenotypic changes in their lung endothelium when obese (Supplementary Fig. 5). Collectively, these findings suggest that low serum adiponectin levels might serve as a marker for identifying individuals at risk for developing ARDS^39^ and that it may have a causal role in determining the susceptibility to this condition. Human studies will be required to establish the role, if any, of serum adiponectin testing in the risk assessment for ARDS.

In our model systems, repletion of adiponectin protected from ALI in obese mice. Although our studies did not elucidate the precise mechanism(s) by which adiponectin mediates these protective effects, we postulate that both direct and indirect effects of adiponectin on the vascular endothelium may be important: direct effects may include adiponectin’s ability to block neutrophil rolling along the endothelium and to inhibit NFkB-mediated transcriptional responses^18^. Indirect effects of adiponectin include its lipid and glucose lowering properties that might, in turn, affect endothelial cell functions through altering the blood environment. Notably, we observed a decrease in serum lipids after adiponectin gene therapy in our obese mice. Whether altered lipid levels contribute to pulmonary protection from ALI needs to be formally tested.

In conclusion, we have shown that obesity disrupts pulmonary vascular immune functions and alters the expression of endothelial junctional adherens and adhesion proteins. These perturbations are associated with enhanced susceptibility of the pulmonary vasculature to injury. Our findings may have important implications for understanding the pathogenesis of inflammatory vascular diseases of the lung in obese humans. Moreover, our studies provide a rationale for pursuing adipokines, and adiponectin in particular, as prognostic and possibly therapeutic targets in obese individuals at risk for ARDS.

## Materials and Methods

All methods were carried out in accordance with the approved guidelines.

### Animals

Male three-week-old AKR/J and DBA/2J mice were purchased from the Jackson Laboratory (Bar Harbor, ME) and housed in a pathogen-free animal facility at Thomas Jefferson University. Mice were maintained on a standard chow diet (13.5% calories from fat, 58% from carbohydrates, and 28.5% from protein) for 1 week and then switched to a “high fat/western-style” diet (42% calories from fat) for a total of 14 weeks. Lean controls were maintained on a standard chow diet for the entire study period. Body weight was assessed once weekly in all mice while fasting blood glucose levels and glucose tolerance testing were performed on only a subset of mice at 14 weeks. Complete blood count (CBC) was performed using a Hemavet 950 FS automated cell counter (Drew Scientific Inc., Oxford, CT.). Prior to initiating studies, all protocols were approved by the Institutional Animal Care and Use Committee at Thomas Jefferson University.

### Murine Model of Acute Lung Injury (ALI)

ALI was induced by a one-time instillation of lipopolysaccride (LPS, 100 mcg) into posterior oropharyngeal space of anesthesized mice as described previously^16^. Animals were sacrificed 24 hours after LPS administration and blood, bronchoalveolar lavage (BAL) fluid, and lung tissues were harvested for analysis. Lung wet:dry ratio and Evan’s blue dye extravasation were performed as previously described^16^,^40^.

### Analysis of BAL fluid

BAL was performed by cannulating the trachea with a blunt 22-gauge needle and instilling one ml of sterile PBS into the lung. Total cell count in the BAL fluid was determined with a TC20 automated cell counter (Bio-Rad Laboratories, Inc., Hercules, CA) while differential cell counts were performed on cells which were cyto-centrifuged onto glass slides (Fisher Scientific). Total protein concentration in the BAL fluid was determined using the Pierce^TM^ BCA assay kit (Thermo Scientic, Rockford, IL) as previously described^16^.

### Enzyme-linked immunosorbent assay

TNF-α, IL-6, KC, MIP-2, IgM, E-selectin, Leptin, and Adiponectin were quantified using commercially available DuoSet ELISA kits (R&D Systems) according to the manufacturer’s instructions as previously described^23^.

### Echocardiography

Cardiac geometry and function were evaluated using the Vevo 2100 imaging system (VisualSonics, Toronto, Canada)^41^. Heart rate was maintained between 350–500 beats/min by titrating isoflurane anesthesia between 0.5–2% volume-to-volume. Body temperature was regulated throughout the procedure using a thermal heat plate. Left ventricle dimension, percent fractional shortening, left ventricular mass index, anterior wall thickness, posterior wall thickness and relative wall thickness were calculated as previously described^42^. Right ventricular imaging was obtained by short-axis transverse view at the level of aortic valve. All images were digitally recorded and analyses were performed using Vevo 2100-software.

### Invasive hemodynamic measurements

Hemodynamic measurements were performed on anesthetized mice placed in the supine position. Cervical blood vessels were visualized by carefully dissecting away the superficial tissues of the neck. A micro tipped transducer/conductance catheter (1.4 French, Millar SPR-671, TX) was then inserted into the carotid artery or jugular vein and slowly advanced toward the right or left ventricle while continuously monitoring arterial or venous pressures.

### Analysis of Serum Free Fatty acid, Triglyceride and Cholesterol levels

Serum free fatty acid, triglyceride and cholesterol levels were measured using commercially available kits (Biovision, Mountain View, CA) according to the manufacturer’s instructions.

### Gene expression analysis by Real-time PCR

For total lung RNA analysis, cDNA was synthesized from 1 μg of total RNA using iScript™ reverse transcription (Bio-Rad) kit. Expression of VCAM-1, ICAM-1, E-selectin, and the internal control GAPDH mRNA levels were analyzed using real-time RT-PCR on an iCycler thermocycler (Bio-Rad Laboratories). TaqMan assays were from Applied Biosystems (assays on demand); VCAM-1 (Mm01320970_m1), ICAM-1 (Mm00516023_m1), E-selectin (Mm00441278_m1) and GAPDH (4352339E).The relative quantity of target genes were calculated by iCycler iQ Real-Time Detection System software (version 3.0a; Bio-Rad) using the comparative threshold method (ΔΔC_t_) and GAPDH as endogenous control.

### Western blot analysis

Western blot analysis was performed as described previously^43^. In brief, lung tissues were homogenized in ice cold lysis buffer (PBS, 0.5% Triton X-100, pH 7.4) containing protease and phosphatase inhibitors (Roche Complete mini). Lung homogenate was centrifuged (14,000 × g) at 4 °C for 15 min and supernatant was collected for further analysis. Twenty micrograms of protein were loaded onto each well, separated on 10% SDS-polyacrylamide gel and then transferred onto a nitrocellulose membrane (Bio-Rad) using a Bio-Rad Mini-Blot transfer apparatus. Immunoblotting was performed at 4 °C overnight using primary antibodies directed against ICAM-1 (R&D Systems, MN), VCAM-1 (Abcam, Cambridge, MA.), E-selectin (Abcam, Cambridge, MA), VE-cadherin (Cell Signaling, Danvers, MA), β-Catenin (Cell Signaling, Danvers, MA), p-Src (Tyr416) (Cell Signaling, Danvers, MA) and GAPDH (Cell Signaling, Danvers, MA). Membranes were then incubated with a 1:5000 dilution of a secondary antibody (Li-Cor Biosciences, Lincoln, NE) at room temperature for 1 hr. Protein bands were visualized using the Odyssey infrared imaging system (Li-Cor Biosciences, Lincoln, NE).

### Immunohistochemistry

Immunohistochemical staining was performed on de-paraffinized lung sections after antigen retrieval with Retrievagen A (Target Retrieval Solution; Dako, CA) and after quenching endogenous peroxidases with 3% H_2_O_2_. Tissues were then blocked with 2% BSA followed by overnight exposure with primary anti-Gr1 antibody (R&D Systems, Minneapolis, MN). The following morning, slides were washed with PBS and secondary antibody was applied for 1 h at room temperature. Staining was visualized using Vectastain ABC reagent (Vector Laboratories, Burlingame, CA) followed by the addition of 3,39-diaminobenzidine (Vector Laboratories).

### Construction of plasmid DNA

Full length cDNA for adiponectin was cloned from mouse fat (primers were 5′-ATG CTA CTG TTG CAA GCT CT-3′ and 5′-TCA GTT GGT ATC ATG GTA GA-3′) and was sequence verified. The adiponectin cDNA was inserted into the pTarget vector using pTarget™ mammalian expression vector system (Promega, Madison, USA). Amplification of the plasmid DNA and removal of bacterial endotoxin was performed using the Endo Free Plasmid Maxi Kit (Invitrogen, Germany).

### Hydrodynamics-based Adiponectin gene delivery

Adiponectin gene delivery was performed as previously described^44^. Briefly, anesthesized mice were placed in a restraining box and the tail vein was immersed in warm water to induce vasodilation. pTarget-adiponectin (1 μg/g body weight) or control plasmid (pTarget) were injected via the tail vein in saline. At specified time points after plasmid delivery serum was collected for measurement of adiponectin, leptin, cholesterol, triglyceride and free fatty acids.

### Lung endothelial cell isolation

Lungs were dissociated into a single-cell suspension using a mouse lung dissociation kit (Miltenyi Biotec, Bergisch Gladbach, Germany) with the gentle MACSTM dissociator according to the manufacturer’s protocol. Endothelial cells were isolated in a two-step process: first, cells were incubated with Microbeads (Miltenyi Biotec) recognizing CD45 and passed through a column to remove immune cells from the suspension, next, endothelial cells were tagged using Microbeads (Miltenyi Biotec) that bind to CD31 and cell suspensions were passed through a column to isolate endothelial cells by positive selection. The purity of the endothelial cell population was confirmed by flow cytometry as previously described^16^.

### Cell culture

Primary mouse lung microvascular endothelial cells (MLECs) and complete mouse endothelium cell medium were both purchased from Cell Biologics, (Chicago, IL). Cells were maintained in 10-cm plastic dishes pre-coated with Gelatin-Based Coating Solution (Cell Biologics, Chicago, IL). For some experiments, MLECs were cultured with serum from lean or obese mice (10 μl serum/ml complete mouse endothelium cell medium containing 1% FBS). At pre-specified time points, cell lysates were collected for later analysis. All *in vitro* studies were performed using cells from passage 3–4.

### Statistical analysis

Statistics were performed using GraphPad Prism 5.0 software. Two-group comparisons were analyzed by unpaired Student’s t-test and multiple-group comparisons were performed using one-way analysis of variance (ANOVA) followed by Tukey post hoc analysis. Statistical significance was achieved when *P* < 0.05 at 95% confidence interval. No animals were excluded from the analysis.

## Additional Information

**How to cite this article**: Shah, D. *et al.* Obesity-induced adipokine imbalance impairs pulmonary vascular endothelial function and primes the lung for injury. *Sci. Rep.* **5**, 11362; doi: 10.1038/srep11362 (2015).

## Supplementary Material

Supplementary Information

## Figures and Tables

**Figure 1:** Obesity promotes endothelial cell activation in the lung. (**a**) Enzyme-linked immunosorbent assay for E-selectin in the serum of lean and obese mice (n = 8, *p < 0.05 vs. NCD group) at baseline (BSL). (**b**) Transcript levels for ICAM-1, VCAM-1 and E-selectin in the lungs of lean and obese mice (n = 4, *p < 0.05 vs. NCD group) at BSL. (**c**) Western blot analysis for ICAM-1, VCAM-1 and E-selectin in the lungs of lean and obese mice at BSL. Image is representative of two different blots. Densitometry analysis shown below (n = 6, *p < 0.05 and **p < 0.01 vs. NCD group). Full length blots are presented in Supplementary Figure 6. (**d**) Western blot analysis for ICAM-1, VCAM-1 and E-selectin in freshly isolated lung endothelial cells from lean and obese mice. Image is representative of two different blots. Densitometry analysis shown below (n = 4, *p < 0.05 vs. NCD group). Full length blots are presented in Supplementary Figure 7. (**e**) Western blot analysis for VE-cadherin, β-Catenin and pSrc in the lungs of lean and obese mice at BSL. Image is representative of two different blots. Densitometry analysis shown on below (n = 6, *p < 0.05 and **p < 0.01 vs. NCD group). Full length blots are presented in Supplementary Figure 8. (**f**,**g**) Evan’s blue dye extravasation and BAL fluid total protein concentrations in the lungs of lean and obese AKR/J mice (n = 5–8 each group) at BSL. Data are expressed as mean ± SE. The statistical significance was assessed using a Student’s unpaired t test.

**Figure 2:** Serum from obese mice promotes lung endothelial activation. (**a**–**e**) Serum free fatty acid, triglyceride, cholesterol, leptin and adiponectin levels in lean and obese mice (n = 8, (*p < 0.05, **p < 0.01, ***p < 0.001 high fat diet (HFD) vs. normal control diet (NCD) group). (**f**) Western blot analysis for ICAM-1, VCAM-1 and E-selectin expression in primary lung microvascular endothelial cells cultured with serum from lean or obese mice for 24 h. Image is representative of two different blots. Full length blots are presented in Supplementary Figure 9. Densitometry analysis shown below (*p < 0.05 and **p < 0.01 vs. NCD serum). (**g**) Western blot analysis for VE-cadherin, β-Catenin and pSrc in primary lung microvascular endothelial cells cultured with serum from lean or obese mice for 24 h. Image is representative of two different blots. Densitometry analysis shown on right (*p < 0.05 vs. NCD serum). Full length blots are presented in Supplementary Figure 10. Data are expressed as mean ± SE. The statistical significance was assessed using a Student’s unpaired t test.

**Figure 3:** Obesity exacerbates LPS-induced lung inflammation and neutrophil influx. (**a**,**b**) Total and neutrophil cell counts in the BAL fluid of lean and obese AKR/J mice at baseline (BSL) and 24 h after *it.* LPS (n = 8 each group, ***p < 0.001 vs. NCD group). (**c**) Immunohistochemical staining for the granulocyte marker Gr-1 (brown stain) in the lungs of lean and obese mice 24 h after *it.* LPS. Morphometric analysis demonstrates an increase in Gr1(+) cells in the lungs of obese mice 24 h after *it.* LPS (n = 3 each group, *p < 0.05 vs. NCD group). Gr-1(+) cells were not readily detected in the lungs of lean or obese mice at baseline (data not shown). (**d**,**e**) Enzyme-linked Immunosorbent assay (ELISA) for TNF-α and IL-6 in lung homogenate from lean and obese AKR/J mice at baseline and 24 h after *it.* LPS (n = 8 each group, *p < 0.05, **p < 0.01 and ***p < 0.001 vs. NCD group). (**f**,**g**) ELISA for the chemokine KC and MIP2 in lung homogenate from lean and obese AKR/J mice at baseline and 24 h after *it.* LPS instillation (n = 8 each group, *p < 0.05, **p < 0.01 and ***p < 0.001 vs. NCD group). Data are expressed as mean ± SE. The statistical significance was assessed using a Student’s unpaired t test and one-way analysis of variance (ANOVA). NCD stands for normal control diet while HFD stands for high fat diet.

**Figure 4:** Obesity impairs endothelial junction and leads to vascular injury. (**a**) Transcript levels for ICAM-1, VCAM-1 and E-selectin in the lungs of lean and obese mice at 24 h after LPS administration (n = 4, *p < 0.05 and **p < 0.01 vs. NCD group). (**b**) Western blot analysis for ICAM-1, VCAM-1 and E-selectin in the lungs of lean and obese mice 24 h after LPS administration. Image is representative of two different blots. Densitometry analysis shown below (n = 6, *p < 0.05 and **p < 0.01 vs. NCD group). Full length blots are presented in Supplementary Figure 11. (**c**) Western blot analysis for VE-cadherin, β-Catenin and pSrc in the lungs of lean and obese mice 24 h after LPS administration. Image is representative of two different blots. Densitometry analysis shown below (n = 6, *p < 0.05 vs. NCD group). Full length blots are presented in Supplementary Figure 12. (**d**) Lung wet/dry ratio in lean and obese AKR/J mice (n = 5 each group, *p < 0.05 and **p < 0.01 vs. NCD group) at baseline and 24 h after *it.* LPS. (**e**–**g**) Evan’s blue dye extravasation and BAL fluid protein concentrations (Total and IgM) in the lungs of lean and obese AKR/J mice (n = 5–8 each group, *p < 0.05, **p < 0.01 and ***p < 0.001 vs. NCD group) at baseline and 24 h after *it.* LPS. (**h**) Representative sections of H&E stained lungs from lean and obese mice 24 h after it. LPS. Peri-vascular edema (shown as black arrows) was increased in the lungs of obese mice, when compared to lean controls (n = 3 each group). Bars indicate 40 μm. Data are expressed as mean ± SE. The statistical significance was assessed using a Student’s unpaired t test and one-way analysis of variance (ANOVA). NCD stands for normal control diet while HFD stands for high fat diet.

**Figure 5:** Restoration of serum adiponectin levels suppresses endothelial cell activation in the lungs of obese mice. (**a**–**d**) Serum adiponectin, free fatty acid, triglyceride and leptin levels in obese mice 3 days after adiponectin gene delivery (n = 8, *p < 0.05, **p < 0.01 vs. HFD group). (**e**) Increasing serum adiponectin levels decreased expression of ICAM-1, VCAM-1 and E-selectin in the lungs of obese mice. Image is representative of two different blots (n = 6, *p < 0.05 vs. HFD group). Densitometry analysis shown below. Full length blots are presented in Supplementary Figure 13. (**f**) Western blot analysis for VE-cadherin, β-catenin and pSrc in the lungs of lean and obese mice 24 h after LPS administration. Image is representative of two different blots. Densitometry analysis shown below (n = 6, *p < 0.05 vs. HFD group). Full length blots are presented in Supplementary Figure 14. Data are expressed as mean ± SE. The statistical significance was assessed using a Student’s unpaired t test. HFD stands for high fat diet and HFD+APN stands for obese mice treated with adiponectin gene therapy.

**Figure 6:** Restoration of serum adiponectin levels attenuates LPS-induced acute lung injury in obese mice. (**a**) Adiponectin gene delivery decreased TNF-α expression in the lungs of obese mice (n = 8 each group, *p < 0.01 vs. HFD group). (**b**,**c**) Adiponectin gene delivery significantly decreased immune cell influx into the lung 24 h after *it.* LPS (n = 8 each group, *p < 0.05 vs. HFD group). (**d**) Adiponectin gene delivery reduced ICAM-1, VCAM-1 and E-selectin expression in the lung after *it.* LPS. (*p < 0.05, and **p < 0.01 vs. HFD group by densitometry). Image is representative of two different blots. Densitometry analysis shown below. Full length blots are presented in Supplementary Figure 15. (**e**) Adiponectin gene delivery enhanced VE-cadherin, β-Catenin and pSrc expression in the lung after *it*. LPS. (*p < 0.05 vs. HFD group by densitometry). Image is representative of two different blots. Densitometry analysis shown on right. Full length blots are presented in Supplementary Figure 16. (**f**,**g**) Adiponectin gene delivery significantly decreased total and IgM protein concentration in the BAL fluid 24 h *it*. after LPS (n = 6 each group, *p < 0.05 vs. HFD group). H) Representative H&E stained lung sections from LPS-injured obese mice receiving adiponectin or empty vector. Peri-vascular edema was decreased in obese mice that received the gene for adiponectin (n = 3 each group). Data are expressed as mean ± SE. The statistical significance was assessed using a Student’s unpaired t test. HFD stands for high fat diet and HFD + APN stands for obese mice treated with adiponectin gene therapy.
